The article "Drug-Eluting Stents for Acute Coronary Syndrome: A Meta-Analysis of Randomized Controlled Trials" was retracted in 2016. Reason: false authorship.

# Drug-Eluting Stents for Acute Coronary Syndrome: A Meta-Analysis of Randomized Controlled Trials

**DOI:** 10.1371/journal.pone.0072895

**Published:** 2013-09-05

**Authors:** Lishan Wang

**Affiliations:** 1 Bio-X Institutes, Key Laboratory for the Genetics of Developmental and Neuropsychiatric Disorders (Ministry of Education), Shanghai Jiao Tong University, Shanghai, P.R. China; 2 FengHe (ShangHai) Information Technology Co., Ltd, Shanghai, P.R. China; University of Virginia Health System, United States of America

## Abstract

**Background:**

Drug-eluting stents (DES) are increasingly used for treatment of acute coronary syndrome (ACS). However, clinical efficacy and safety of various types of DES is not well established in these subjects. We therefore evaluated clinical utility of second-generation and first-generation DES in patients with ACS by conducting a meta-analysis.

**Methods:**

A search of Medline, Embase, the Cochrane databases, and Web of Science was made. Randomized controlled trials (RCTs) which compared second-generation DES (everolimus-eluting stents [EES] or zotarolimus-eluting stents [ZES]) versus first-generation DES (sirolimus-eluting stents [SES] or paclitaxe-eluting stents [PES]) in patients with ACS and provided data on clinical efficacy or safety endpoints were included. Pooled estimates were calculated using random-effects model.

**Result:**

A total of 2,757 participants with ACS in 6 RCTs were included. Compared with first-generation one, second-generation DES trended to be associated with the decreased incidence of definite or probable stent thrombosis in ACS patients (risk ratio [RR]  = 0.60, 95% confidence intervals [CI] 0.33 to 1.07, p = 0.09). However, the rate of target lesion revascularization (TLR) significantly increased in second-generation DES (RR = 2.08, 95%CI 1.25 to 3.47, p = 0.005). There were no significant differences in the incidence of major adverse cardiac events (MACEs), all-cause death, cardiac death, and recurrent myocardial infarction between the two arms (all p>0.10). The second-generation EES showed a tendency towards lower risk of MACEs (p = 0.06) and a beneficial effect on reducing stent thrombosis episodes (p = 0.009), while the second-generation ZES presented an increased occurrence of MACEs (p = 0.02) and TLR (p = 0.003).

**Conclusion:**

Second-generation DES, especially EES, appeared to present a lower risk of stent thrombosis, whereas second-generation ZES might increase the need for repeat revascularization in ACS patients. During coronary interventional therapy, DES class should be adequately considered in order to maximize clinical benefit of DES implantation in these specific subjects.

## Introduction

Drug-eluting stents (DES) are increasingly used for treatment of acute coronary syndrome (ACS). Previous randomized controlled trials (RCTs) and meta-analysis have demonstrated that DES were superior to bare-metal stents in minimizing the occurrence of stent restenosis and reducing the need for revascularization in patients with ACS [1], [2], [3], [4], [5], which was the major drawback of percutaneous coronary interventions (PCI) in bare-metal stents era. In patients in stable condition the newer second-generation DES, eluting with everolimus (EES) or zotarolimus (ZES), has shown promise in improving further the clinical outcomes compared with the first-generation sirolimu- or paclitaxe-eluting stent (SES or PES) [6], [7], [8]. However, the issue that whether clinical utility of various types of DES in treating ACS settings with the higher possible thrombotic coronary lesions is identical remains uncertain. To date there is a limited number of registry studies and RCTs comparing the second-generation versus first-generation DES in ACS patients and delivering conflicting results. Korea Acute Myocardial Infarction Registry (KAMIR) study showed that the first-generation SES had the lower 1 year incidences of major adverse cardiac events (MACEs) and target lesion revascularization (TLR) than the second-generation ZES in patients with ST-segment elevation myocardial infarction undergoing primary PCI [9]. However, the benefit of the first-generation DES was not shown in an early small-scale study [10] and a randomized trial [11]. In contrast, the second-generation EES appeared to be associated with lower incidences of MACEs [12] and definite and/or probable stent thrombosis in patients with ST-segment elevation myocardial infarction [13]. These inconsistent findings confused interventional cardiologists' stent selection decisions beyond consideration of characteristics of device performance. As thus, here we conducted a meta-analysis of RCTs to evaluate the clinical outcomes of ACS patients treated with the second- versus the first-generation DES.

## Materials and Methods

### Eligible criteria

The clinical studies were eligible for inclusion if 1) study design involved patient randomization; 2) they compared second-generation DES (EES or ZES) versus first-generation DES (SES or PES) in patients with ACS (unstable angina, non-ST segment elevation acute myocardial infarction, and ST segment elevation acute myocardial infarction); 3) the information on clinical efficacy or safety endpoints (e.g. MACEs, all-cause death, cardiac death, recurrent myocardial infarction, TLR, or definite and/or probable stent thrombosis) was available; 4) follow-up duration was no less than 6 months. We restricted our analyses to the DES approved by the US Food and Drug Administration (FDA). Trials would be excluded if the data on patient and procedural characteristics was not available, and post-hoc analyses of RCTs were also excluded.

### Study identification

We performed an electronic search of Medline, Embase, the Cochrane Central Register of Controlled Trials, the Cochrane Database of Systematic Reviews, and ISI Web of Science until December 2012 for the eligible trials. Complex search strategies were formulated using the following terms: *everolimus-eluting stent, zotarolimus-eluting stent, second-generation eluting stent, sirolimus-eluting stent, paclitaxel-eluting stent, first-generation eluting stent, unstable angina, acute myocardial infarction, and acute coronary syndrome*. We also checked the references and citations of the eligible studies from the potential eligible articles to ensure that no clinical trials were missed. The search was restricted to English-language literature.

### Study enrollment, data collection, and quality assessment

Two investigators (W.L., Z.W.) assessed trial eligibility using predefined eligibility criteria in duplicate and independently. The data, such as participant characteristics, lesion and procedural characteristics, and follow-up duration from each study, were extracted. The occurrence of clinical outcomes was also recorded. Any disagreements were resolved through consensus. Also all the eligible trials were assessed by the following quality criteria recommended by the Cochrane Collaboration: sequence generation of the allocation; concealment of allocation; blinding of participants, personnel, and outcome assessors; use of intention to treat analysis; description of withdrawals and dropouts. A numerical score between 0 and 5 was assigned as a measure of study design and reporting quality with 0 being the weakest and 5 designated the strongest, based on the validated scale put forward by Jadad and colleagues [14].

### Statistical analyses

Treatment effects were reported as risk ratio (RR) with 95% confidence intervals (CI). Pooled estimates were calculated with random-effects model. For studies with no event of interest in a treatment group, 1.0 was added to all cells for continuity correction [15]. Statistical homogeneity was quantified with the I^2^ statistic with a scale of 0% to 100% (>75% represented very large between-study inconsistency) [16]. Subgroup analysis was performed to test the potential influence of clinical factors including ACS classification, mean age, time from pain to angioplasty, percentage of TIMI grade 0/1, type of DES, stent length, stent size, and follow-up duration. For verification of the robustness of the results, sensitivity analyses were conducted by alternatively using fixed-effect model, and by omitting each trial at a time from analysis and then computing overall estimates for the remaining studies. The potential publication bias was qualitatively assessed using funnel plot method. The significance level was set at p<0.05. The pooling analyses were performed using Review Manager 5.1 software (Cochrane Collaboration, Copenhagen, Denmark). The present work was performed as the guidelines proposed by Preferred Reporting Items for Systematic Reviews and Meta-Analyses (PRISMA) (Checklist S1).

## Results

Results from our literature search were detailed in Figure 1. Briefly, our initial search yielded 880 potential literature citations from the electronic databases. Of them, 734 were excluded by removing duplicate literatures and through review of citations. Abstracts from 146 articles were reviewed and an additional 79 trials were excluded, leaving 67 studies for full publication review. Thereafter 61 were excluded (43 were non-randomized studies, 12 used DES which were not approved by FDA, 3 had no data on clinical characteristics, 1 was post-hoc analysis of RCTs, 2 were pooled analysis of RCTs) and no additional relevant study was identified from the references and citations of eligible articles. Finally, 6 studies were found to conform to the predefined inclusion criteria [11], [12], [13], [17], [18], [19].

**Figure 1:** Flow chart of studies selection. DES  =  drug-eluting stents; RCTs  =  randomized controlled trials; FDA  =  the US Food and Drug Administration.

The demographic, clinical, and procedural characteristics of the 6 trials were shown in Table 1 and Table 2. A total of 2,757 participants with ACS were enrolled in the meta-analysis. Among them 1,302 were randomly allocated to receive second-generation DES implantation and 1,455 to receive first-generation DES treatment. Of the enrolled 6 trials, two [11], [17] were three-arm trials (ZES vs. PES vs. SES), but the rest were two-arm trials (two [12], [13] for EES vs. SES; two [18], [19] for ZES vs. SES). Five [11], [12], [13], [17], [18] focused on patients with acute myocardial infarction, and one [19] on unrestricted ACS in which only 16.2% ST-segment elevation acute myocardial infarction was involved. Four trials reported 30 day follow-up clinical outcomes [11], [12], [13], [17]; 5 reported 6–12 month data [11], [12], [13], [17], [18]; and 2 reported 18 month data [17], [19]. The majority of participants was male and the mean age ranged from 59.7 years to 65.3 years. Total stent length per patient ranged from 22.5 mm to 31.6 mm and mean size of stents from 3.14 mm to 3.27 mm. All of the enrolled patients received dual antiplatelet therapy no less than 12 months or to the end of the follow-up. Additionally, the level of evidence for each article was graded with a score of 3 to 4 according to the Jadad quality score (Table S1).

**Table 1:** Baseline patient characteristics of randomised controlled trials included in the meta-analysis.

Study, year	No. enrolled, randomization ratio	Comparisons	Study design	Mean age	Male %	Diabetes, %	Current smoker, %	Pain to angioplasty, h	NS TEACS, %	STEAMI, %	Target vessel (LAD/LCX/ RCA/LM), %	Primary end points	Follow-up methods	Follow-up duration
KOMER, 2011	611, 1:1:1	ZES vs. PES vs. SES	single-blind, multicentre	59.7	79	20.8	54.8	5.3	0	100	53.8/6/37.2/0	MACEs	Angiography	30d, 12m,18m
Sawada T, 2012	35, 2:1	EES vs. SES	single-blind, single center	65.3	78.8	42.4	42.4	NA	0	100	60.6/0.03/37.7/0	NIT and stent thrombosis	OCT, angioscopy, angiography	30d, 7m
SEZE, 2012	121, 1:1	ZES vs. SES	single-blind, multicentre	60.9	81	22.3	53.8	5.3	0	100	58/9/33/0	Late lumen loss	Angiography, IVUS	12m
SORT OUT III ACS, 2012	1052, 1:1	ZES vs. SES	open-label, multicentre	63.1	73.1	13.6	38.5	NA	83.8	16.2	40.95/27.25/2 9.95/1.65	MACEs	Angiography	18m
XAMI 2012	625, 2:1	EES vs. SES	single-blind, multicentre	61.5	73.7	9.7	54.7	2.85	4	96	40.1/19/40.4/0.2	MACEs	Angiography	30d, 12m
ZEST AMI, 2009	328, 1:1:1	ZES vs. PES vs. SES	single-blind, multicentre	59.7	82.3	25.9	56.7	4.75	0	100	46.3/11.6/42.1/0	MACEs	Angiography	30d, 12m

MACEs was defined as cardiac death, recurrent myocardial infarction, and target vessel or lesion revascularization. EES  =  everolimus-eluting stents. IVUS  =  intravascular ultrasound; LAD  =  left anterior descending artery; LCX  =  left circumflex artery; LM  =  left main artery; MACEs  =  major adverse cardiac events; NA  =  not available; NIT  =  neointimal thickness; NSTEACS  =  non-ST-segment elevation acute coronary syndrome; OCT  =  optical coherence tomography; PES  =  paclitaxel-eluting stents. RCA  =  right coronary artery; SES  =  sirolimus-eluting stents; STEAMI  =  ST-segment elevation acute myocardial infarction; ZES  =  zotarolimus-eluting stent.

**Table 2:** Baseline lesion and procedural characteristics.

Study, year	Reference vessel diameter, mm	Lesion length, mm	No. of lesions per patient	No. of stents per patient	Total stent length per patient, mm	Stent size (mm)	Multivessel disease	Initial TIMI grade flow, 0/1/2/3, %	Final TIMI grade flow after procedure, 0/1/2/3, %	Max inflation pressure, atm	DAPT durati on, m	Use of glycoprotein IIb/IIIa inhibitors, %
KOMER, 2011	2.97	19.5	1.0	1.2	24.1	3.27	42.9	54.3/11.3/16.5/17.9	0/0.1/6.2/93.7	NA	≥12	25
Sawada T, 2012	2.94	NA	NA	NA	22.5	3.14	0	90.9/0/9.1/0	NA	17.8	7	0
SEZE 2012	2.79	23.4	NA	1.15	28.6	3.16	67	63/7.5/11.5/18	0/0/6.5/93.5	15.5	12	12.4
SORT OUT III ACS, 2012	NA	NA	1.42	NA	28.1	3.2	NA	NA	NA	NA	12	22.15
XAMI 2012	NA	NA	NA	1.35	26	NA	47.3	55.4/6.1/17.1/21.4	NA	NA	12	75.6
ZEST AMI 2009	2.96	27.11	1.22	1.51	31.6	3.25	45.1	58.5/10.1/15.5/15.9	0.3/0.6/10.3/88.8	15.2	≥12	19.8

DAPT  =  dual antiplatelet therapy; NA  =  not available; TIMI  =  Thrombolysis In Myocardial Infarction.

Meta-analytic pooling for the incidence of MACEs, all-cause death, and cardiac death showed that the second-generation DES did not provide a greater advantage compared with the first-generation DES in ACS patients (MACEs: RR = 1.13, 95% CI 0.73 to 1.76, p = 0.53, I^2^ = 57%, Figure 2A; all-cause death: RR = 0.88, 95% CI 0.56 to 1.38, p = 0.59, I^2^ = 57%, Figure 2B; cardiac death: RR = 0.82, 95% CI 0.35 to 1.92, p = 0.65, I^2^ = 12%, Figure 2C). Moreover, second-generation DES did not show the superiority in lowering the risk of recurrent myocardial infarction (RR = 0.83, 95% CI 0.27 to 2.61, p = 0.75, I^2^ = 53%, Figure 3A). Notably, the risk for TLR in ACS patients receiving second-generation DES treatment was over 2 times higher than the first-generation DES (RR = 2.08, 95%CI 1.25 to 3.47, p = 0.005, I^2^ = 0%, Figure 3B). Conversely, the second-generation DES trended to be associated, albeit nonsignificantly, with decreased incidence of definite or probable stent thrombosis (RR = 0.60, 95%CI 0.33 to 1.07, p = 0.09, I^2^ = 15%, Figure 3C).

**Figure 2:** Pooled risk ratios of second-generation versus first-generation drug-eluting stents for acute coronary syndrome for major adverse cardiac events (A), all-cause mortality (B), and cardiac death (C). CI  =  confidence intervals; DES = drug-eluting stents; M–H  =  Mantel-Haenszel.

**Figure 3:** Pooled risk ratios of second-generation versus first-generation drug-eluting stents for acute coronary syndrome for recurrent myocardial infarction (A), target lesion revascularization (B), and definite or probable stent thrombosis (C). Abbreviations as Figure 2.

In addition, in acute myocardial infarction (AMI) subgroup, there were no significant differences in the occurrence of MACEs and TLR between the two arms (Table 3). Nevertheless, compared with the first-generation DES, the second-generation DES might dramatically lower the risk of stent thrombosis by 54% (RR = 0.46, p = 0.01). However, when the analysis was restricted to unselected ACS patients, in which only one study (SORT OUT III ACS trial [19]) was enrolled, pooled results showed that the second-generation DES was inferior to the first-generation one in reducing the incidence of MACEs (p = 0.02) and TLR (p = 0.01). Nevertheless, the second-generation DES did not increase the risk of stent thrombosis compared with the first-generation one (p = 0.48). In ZES subgroup the second-generation DES showed an increased occurrence of MACEs (RR = 1.45, p = 0.02) and TLR (RR = 2.31, p = 0.003), while in EES subgroup a tendency to lower the risk of MACEs (RR = 0.55, p = 0.06) and a benefit in reducing stent thrombosis episodes were found (RR = 0.39, p = 0.009). With the prolongation of follow-up duration, the unfavorable effects of the second-generation DES on MACEs and TLR became statistically significant at 18 months post stent implantation (MACEs: RR = 1.62, p = 0.01; TLR: RR = 2.66, p = 0.002). Nevertheless, the second-generation DES showed a tendency toward lowering the risk of stent thrombosis at 30 days (RR = 0.35, p = 0.06), and the benefit became significant statistically at 6 to 12 months after stent implantation (RR = 0.48, p = 0.01). Moreover, in ACS patients with lower TIMI grade (TIMI 0/1) the second-generation DES might show the more beneficial effect on lowering the risk of stent thrombosis in comparison to the first-generation one (RR = 0.36, p = 0.02). In addition, time from symptom to angioplasty had little impact on the above clinical endpoints (Table 3).

**Table 3:** Subgroup analyses based on the data on MACEs, TLR, and stent thrombosis.

	MACEs			TLR			Stent thrombosis		
Subgroups	No. of studies	RR (95% CI)	*P* value	No. of studies	RR (95% CI)	*P* value	No. of studies	RR (95% CI)	*P* value
Study on AMI	4	0.97 [0.61, 1.54]	0.90	4	1.92 [0.88, 4.15]	0.10	5	0.46 [0.26, 0.83]	0.01
Study on unclassified ACS	1	1.76 [1.11, 2.80]	0.02	1	2.45 [1.22, 4.93]	0.01	1	1.51 [0.48, 4.73]	0.48
Age ≥60	3	0.98 [0.45, 2.13]	0.95	4	1.88 [1.07, 3.28]	0.03	4	0.58 [0.27, 1.22]	0.15
Age <60	2	1.36 [0.85, 2.20]	0.20	1	3.42[1.01,11.56]	0.05	2	0.54 [0.08, 3.53]	0.52
Pain to angioplasty>5h	2	1.17 [0.69, 1.99]	0.56	2	2.10 [0.78, 5.63]	0.14	2	0.86 [0.28, 2.61]	0.79
Pain to angioplasty<5h	2	0.85 [0.35, 2.07]	0.73	1	1.37 [0.27, 7.01]	0.70	2	0.38 [0.13, 1.14]	0.08
TIMI 0/1≥70%	1	0.89 [0.37, 2.15]	0.79	2	1.07 [0.34, 3.35]	0.91	2	0.36 [0.15, 0.84]	0.02
TIMI 0/1<70%	3	1.00 [0.54, 1.83]	0.99	2	2.47 [0.93, 6.55]	0.07	3	0.59 [0.26, 1.31]	0.19
EES	1	0.55 [0.29, 1.03]	0.06	2	1.06 [0.26, 4.26]	0.94	2	0.39 [0.19, 0.79]	0.009
ZES	4	1.45 [1.06, 1.98]	0.02	3	2.31 [1.34, 3.99]	0.003	4	0.97 [0.45, 2.09]	0.93
30 day follow-up	3	0.73 [0.40, 1.35]	0.32	3	0.82 [0.17, 3.96]	0.80	4	0.35 [0.12, 1.04]	0.06
6–12 month follow-up	4	0.95 [0.61, 1.49]	0.83	4	1.58 [0.72, 3.46]	0.25	5	0.48 [0.26, 0.86]	0.01
18 month follow-up	2	1.62 [1.11, 2.37]	0.01	2	2.66 [1.45, 4.88]	0.002	2	1.23 [0.54, 2.79]	0.63

ACS  =  acute coronary syndrome; AMI  =  acute myocardial infarction; CI  =  confidence intervals; EES  =  everolimus-eluting stents; MACEs  =  major adverse cardiac events; RR  =  risk ratios; TIMI  =  Thrombolysis In Myocardial Infarction; TLR  =  target lesion revascularization; ZES  =  zotarolimus-eluting stent.

In sensitivity analysis, when the XAMI study [12] was omitted from the analysis on MACEs, and the SORT OUT III ACS study [19] from TLR and stent thrombosis, the corresponding original results were reversed (MACEs: RR = 1.45, 95%CI 1.06 to 1.98, p = 0.02, I^2^ = 0%; TLR: RR = 1.73, 95%CI 0.83 to 3.64, p = 0.15, I^2^ = 0%; stent thrombosis: RR = 0.46, 95%CI 0.26 to 0.83, p = 0.01, I^2^ = 0%). Except for the process, omission of each trial one at a time from the analysis or alternatively using fixed-effect model did not have any relevant influence on other overall results in the meta-analysis. Funnel plots were performed for all outcomes and did not show symmetry (Figure S1), suggesting that there exist the substantial publication bias in the meta-analysis.

## Discussion

The present study, to our knowledge, was the first meta-analysis based on the currently available data from RCTs to comparing the clinical values of second-generation versus first-generation DES in patients with ACS. It revealed that ACS subjects treated with the second-generation DES had the similar incidences of MACEs, all-cause death, cardiac death, and recurrent myocardial infarction as those treated with the first-generation DES. However, the second-generation DES was associated with increased risk of repeat revascularization in comparison to the first-generation DES, with the relative risk of TLR of 2.08. Nevertheless, the second-generation DES had a trend toward lower the risk of definite or probable stent thrombosis in overall ACS patients. And the second-generation DES reduced the incidence of stent thrombosis by 54% in patients with acute myocardial infarction. Second-generation ZES might be associated with increased occurrence of MACEs and TLR. Conversely, in patients with acute myocardial infarction, receiving EES implantation, or the lower TIMI grade, the second-generation DES might be the more beneficial in reducing the risk of stent thrombosis than the first-generation one.

Newer second-generation DES was primarily conceived to further improve clinical utility of DES on the basis of first-generation one. Unfortunately, the current study did not show the differences in reducing the incidences of MACEs, all-cause mortality, cardiac death, and recurrent myocardial infarction between the two generations DES in ACS patients. Nevertheless, the overall results in the current study showed that the incidences of the above clinical outcomes were low in both arms. These findings may also reflect the progress over the last few years in ACS patient treatment.

Unexpectedly, the TLR rate in ACS patients undergoing the second-generation DES implantation was higher than that receiving first-generation DES. Of note, of 5 trials enrolled in the analysis of the clinical endpoint, two showed the superiority of first-generation DES [17], [19], and the other 3 did not present intergroup differences. Both KOMER trial [17] and SORT OUT III ACS trials [19] compared clinical efficacy and safety of second-generation ZES versus first-generation SES or/and PES in ACS patients. The two studies consistently demonstrated ZES did not have the superiority and even presented the inferiority in reducing the risk of repeat revascularization to the first-generation DES. Furthermore, the ENDEAVOR III study [20], a prospective, randomized, single-blinded multicenter trial, comparing ZES and SES in patients with stable coronary disease undergoing elective PCI, also indicated that ZES was associated with significantly higher late lumen loss and binary restenosis at 8 month angiographic follow-up. Based on these findings, we presumed that the use of ZES might be the major cause responsible for the unfavorable overall result on TLR. Indeed, when the analysis was restricted to subjects receiving ZES implantation, it showed that the use of the second-generation DES was associated with the higher incidence of TLR. Nevertheless, it was notable that the second-generation ZES included in the meta-analysis has a phosphorylcholine coating polymer that is a synthetic copy of the predominant phospholipid in the outer membrane of red blood cells. The unfavorable finding was not extrapolated automatically to the newer generation of ZES, such as Endeavor Resolute DES, which uses a proprietary new biocompatible polymer called BioLinx. Recently a clinical study [21], comparing the long-term clinical outcomes of the two ZES, indicated that Endeavor Resolute ZES significantly reduced the angiographic in-stent late lumen loss and had a lower 2 year incidence of TLR in patients with coronary heart disease. However, compared with the first-generation DES, the use of the second-generation EES in ACS settings did not provide a significant impact on this clinical endpoint. That is to say, among the second-generation DES, EES should be recommended with priority when the rate of repeat revascularization was regarded as prime target of coronary interventional therapy in ACS patients undergoing PCI.

The propensity for stent thrombosis following first-generation DES implantation after discontinuation of dual antiplatelet therapy has raised safety concerns [22], [23]. Recently a pooled patient-level meta-analysis demonstrated that among patients with ST-segment elevation ACS undergoing primary PCI, the first-generation DES (SES and PES) are associated with the increased risk of very late stent thrombosis and recurrent myocardial infarction compared with bare-metal stents [24]. The development of newer second-generation DES aims mainly to address the issue. A comprehensive network meta-analysis by Palmerini T et al. [25], in which 50,844 patients with unclassified coronary heart diseases were enrolled, showed that the second-generation DES, EES but not ZES, had the lower rate of stent thrombosis within 2 years of implantation than bare-metal stents and first-generation DES. The beneficial effect of EES was also confirmed by another small-scale meta-analysis performed by Alazzoni A et al [26]. However, another meta-analysis of 19 trials including 16,924 unrestricted coronary artery disease subjects did not find the differences in stent thrombosis between the overall second-generation DES and the overall first-generation those during the first year after stent implantation [27]. Unfortunately, these previous consistently focused on the patients with unrestricted coronary heart diseases and did not further perform a pooled analysis on the specific subsets. As thus, safety value of second-generation DES in patients with coronary artery diseases, especially with ACS, was yet not well established. The current meta-analysis investigated the issue and showed a beneficial tendency of the second-generation DES toward lowering the incidence of stent thrombosis compared with the first-generation DES. Moreover, after omitting the SORT OUT III ACS study [19] from the pooling analysis, the intergroup difference became significant. As thus, the original nonsignificant difference might be mainly caused by the enrollment of SORT OUT III ACS study in the meta-analysis. Causally, clinical design of SORT OUT III ACS study differed from that of the others included in the meta-analysis. The high percentage of patients with non-ST segment elevation ACS (83.8%) was recruited in the trial [19]. Non-ST segment elevation ACS was characterized by lower possible thrombotic coronary lesions than ST-segment elevation ACS. That is to say, in terms of lowering the risk of stent thrombosis the second-generation DES might have the more superiority in patients with higher possible thrombotic lesions. Indeed, in acute myocardial infarction subgroup we did find the benefit associated with second-generation DES implantation. Notably, the significant reduction in the occurrence of stent thrombosis was achieved under dual antiplatelet therapy with recommended duration by corresponding clinical guidelines. It was highly commendable for second-generation DES to provide an additional benefit.

Methodologically, the use of random-effect model and relatively low statistical heterogeneities among the included trials might ensure the robustness of conclusions from the current study. Moreover, major results in the present study were further confirmed with sensitivity analyses. However, due to the limited sample size, the findings in the subgroup analyses, especially in the EES subgroup, were not solid enough and should be interpreted with caution. Larger-scale studies will be needed to further verify the findings and conclusions in the subgroup analyses of the current study. In addition, the other limitation of our study was that there existed a substantial publication bias which might influence the overall results. As thus, the publication of negative data should be encouraged to elaborate the true effects of the second-generation DES on the ACS subjects.

In summary, this meta-analysis based on the currently available data from RCTs did not show significant differences in the incidence of MACEs, all-cause death, cardiac death, and recurrent myocardial infarction between the second-generation and the first-generation DES. Nevertheless, the second-generation DES, especially EES, appeared to present a lower risk of stent thrombosis in ACS patients, especially in acute myocardial infarction. However, the second-generation DES, mainly referring to ZES, seemed to increase the need for repeat revascularization compared with the first-generation one. Therefore, in process of interventional therapy for these specific subjects, DES class and ACS classification should be adequately considered in order to maximize clinical benefit of DES implantation.

## Supporting Information

Figure S1 **Publication bias analysis using funnel plot method**.
(TIF)

Table S1 **Quality assessment of the enrolloed trials**.
(DOC)

Checklist S1 **Preferred Reporting Items for Systematic Reviews and Meta-Analyses (PRISMA) checklist**.
(DOC)
